# Expression of serum microRNA-378 and its clinical significance in renal cell carcinoma

**DOI:** 10.1590/1678-4685-GMB-2016-0121

**Published:** 2017

**Authors:** Lixin Shi, Lei Zhang, Chunyang Wang, Shengkun Sun, Xiyuan Cao, Xu Zhang

**Affiliations:** 1 Department of Urology, PLA General Hospital, Beijing, China; 2 Institute of Basic Medicine, Military Medical Science Academy of the PLA, Beijing, China

**Keywords:** Renal cell carcinoma, microRNA 378, diagnosis, patients, AUC

## Abstract

Studies have demonstrated that miRNA-378 is expressed in various malignant tumors. In the present study, we aimed to explore the expression of serum miRNA-378 and its clinical significance in renal cell carcinoma (RCC) patients. A total of 75 RCC patients, 63 renal cysts (RC) patients and 75 healthy controls were selected. The miRNA-378 level in RCC and RC groups was significantly higher than in healthy control group, with RCC group having the highest level. The miRNA-378 levels were significantly decreased within the same group after surgery. When compared with healthy controls, RC group had higher levels but not significantly (p > 0.05) while levels in RCC group were significantly higher (p < 0.05). miRNA-378 expression was correlated with clinical stage and differentiation degree, but not correlated with patient's age, gender, surgical strategy and tumor diameter. The AUC of miRNA-378 was 0.896, 95% confidence interval was 0.847 to 0.945, and AUC hypothesis testing was statistically significant (p < 0.001, RCC vs healthy control). miRNA-378 shows potential in the diagnosis and prediction of postoperative curative effect of renal cell carcinoma, but further studies with lager samples are needed.

## Introduction

Renal cell carcinoma (RCC) is the most common space-occupying lesion in adult kidney. RCC accounts for about 3% of all tumors, and the mortality rate reaches 40% (Franceschi and Wild, 2013; Tan *et al.*, 2015). There is no typical clinical symptom at the early stages and most RCCs are diagnosed at late stages, with symptoms including intermittent hematuria, low back pain, abdominal mass, large tumor area and even with distant metastasis (Golan and Eggener, 2015). RCC is not sensitive to radiotherapy and chemotherapy, and its prognosis is unfavorable (Golan and Eggener, 2015). Although surgical resection is the best treatment currently, relapse still occurs in 20 to 40% of patients. Finding early tumor markers and evaluating their clinical curative effect on RCC have become extremely urgent and important.

MicroRNAs (miRNAs) are non-coding small RNA molecules that contain a loop-stem structure. These miRNAs regulate cell growth and differentiation, and play important roles in the process of life and the development of disease (Cheng *et al.*, 2015; Das *et al.*, 2014; Duan *et al.*, 2014). Studies indicate that miRNAs are closely related to the occurrence and development of tumors (Warnecke-Eberz *et al.*, 2015; Wong *et al.*, 2011; Ye *et al.*, 2013). It has been reported that miRNAs play an important role in the regulation of tumor in prostate, lung, breast and colon cancers. In addition, miRNAs also play important roles in the pathogenesis of RCC (Fedorko *et al.*, 2015; Lin *et al.*, 2010). Wulfken *et al.* (2011) indicated that circulating miR-1233 could serve as a potential biomarker for RCC patients(Wulfken *et al.*, 2011). MiRNA expression profiling has found a number of specific miRNAs in RCC, which mainly act through regulating the balance between cancer genes and tumor suppressor genes (Huang *et al.*, 2014; Juan *et al.*, 2010).

Studies have demonstrated that miRNA-378 is expressed in various malignant tumors, and is related to the survival, migration, invasion, angiogenesis and growth of tumor cells (Chen *et al.*, 2012; Deng *et al.*, 2013; Lee *et al.*, 2007). Reports have shown that miRNA −378 is expressed abnormally in serum of RCC patients, however, the results were inconsistent. Fedorko *et al.* (2015) reported that significantly increased serum levels of miR-378 enabled to clearly distinguish RCC patients and healthy controls. Wang *et al.* (2015a) reported that plasma miR-378 was markedly decreased in patients with RCC, even in those with stage I disease, compared with the non-cancer controls (p < 0.01)(Fedorko *et al.*, 2015; Wang *et al.*, 2015a). In this study, we detected the expression of miRNA-378 in RCC patients from North China, aiming to clarify the role of miRNA-378 in RCC, and investigate its diagnostic feasibility.

## Patients and Methods

### Patients

All procedures performed in human participants were in accordance with the ethical standards of the PLA General Hospital, and complied with the Declaration of Helsinki and its later amendments or comparable ethical standards. All subjects signed a form of informed consent.

In this study, three groups were recruited: primary renal cell carcinoma (RCC) patients, simple renal cyst (RC) patients, and healthy controls. The RCC and RC patients were all recruited from the hospital clinic, had received surgical resection at our department, and their resected tissues were confirmed by pathological examination. Healthy controls were adults in the outpatient physical examination clinic. The age of patients and controls ranged from 18 to 68.

### Blood sample collection

For RCC and RC patients, blood samples were collected at two time points: before surgery and six months after surgery. The fasting serum samples of healthy controls were collected during their physical examination. A total of 3 mL blood samples were taken in SSTII advance tubes (Becton Dickinson, UK) and preserved at 4 °C in a refrigerator for 1 h. The blood samples were centrifuged for 3 min at 500 rpm, the upper level of serum was transferred to a 1.5 mL Eppendorf tube without RNase. Phenol/chloroform were used for deproteinization, ethanol was used to precipitate RNA, and DEPC water was added to dilute the RNA. The overall quality of an RNA preparation was assessed by electrophoresis on a denaturing agarose gel, and purity of extracted RNA was tested by UV spectrophotometry. The OD260/OD280 ratio value should be greater than 1.8.

Computer tomography or ultrasonography and (or) chest X-ray examination were performed to assess tumor recurrence in postoperative RCC patients once a month for six months. The imaging or endoscopic examination indicated recurrence of primary tumor site; regional or distant lymph node metastasis can be considered as recurrence after tumor resection. The follow-up of this study ended in April 2016.

### RT-PCR for miRNA-378

The total serum miRNA was extracted by the microRNA Extraction Kit (miRNeasy Mini Kit, Qiagen, Hamburg, Germany). The reverse transcription polymerase chain reaction (RT-PCR) method was used to measure miRNA-378 levels. The RT-PCR assays were done in a TIANGEN Biotech system (Beijing) in a total volume of 20 μL composed of: 10 μL 2x microRNA premix regent, 0.4 μL self-contained primer, 2 μL RT reaction product, 0.4 μL reverse primer, and 7.2 μL of DEPC water. As intercalating dye, 20xSYBR Green I was used (TIANGEN Biotech, Beijing, CHN) and assays were run in a CFX96 Touch Real-Time PCR Detection System (BioRad, Hercules, CA, USA) for quantitative measurement with the following conditions: 95 °C for 10 min, 95 °C for 15 s, 60 °C for 1 min (40 cycles). The relative expression of miRNA-378 was calculated according to (Schmittgen and Livak 2008): F = 2^–Δct^, Δct = ctmiRNA-378 - ctmiRNA-U6. MIR378 (MIMAT0000731) miRNA qPCR Primer Pairs was purchased from OriGene Technologies Inc (Rockville, MD, USA), with the following primer sequence: forward 5’ CTCCTGACTCCAGGTCCTGT3’, and reverse 5’ GCCTTCTGACTCCAAGTCCA 3’. U6 primers were synthesized by Life Technology (Shanghai, China): RT 5’CGCTTCACGAATTTGCGTGTCAT3’U, and forward 5’GCTTCGGCAGCACATATACTAAAAT3’

### Statistical analysis

The relative expression levels of miRNA-378 were reported as the means and standard deviations. The data were analyzed by SPSS 17 software (IBM, Chicago, IL, USA) with Wilcoxon rank sum test and H Kruskal-Wallis rank sum test. The sensitivity and specificity of miRNA-378 were calculated by ROC curve (AUC) based on the data collected from healthy controls and RCC patients; Graphpad Prism 5.0 software (GraphPad Software, San Diego, USA) was used for ROC curve analysis. A p < 0. 05 was considered as statistically significant.

## Results

### Demographic data

From April 2011 to December 2014, a total of 75 RCC patients and 63 RC patients were selected. In addition, blood samples from 75 healthy controls were collected. The demographic data of these patients are listed in Table 1. Six patients were lost to follow up. The follow up time of RCC patients ranged from 8 to 61 months with average of 38.6 ± 16.2 months. A total of 18 patients had recurrence during the follow-up, 8 of them relapsed within 1 year after surgery; 4 within 1 to 3 year after surgery and 6 within 3 to 5 years.

**Table 1:** Demographic data of selected subjects.

	Healthy	RCC	RC
Case number	75	75	63
Age	62.07 ± 3.21	59.72 ± 2.96	61.03 ± 3.67
Gender (M/F)	40/35	48/37	42/21
Tumor location (left/ right)	–	39/36	
Tumor diameter (mm)	–	2.7 ± 0.8	
Follow up period (month)	–	38.6 ± 16.2	1.5 ± 1.2

### miRNA-378 expression before surgery

We first compared the miRNA-378 expression in healthy controls, and in RC and RCC patients. As shown in Figure 1, the expression of miRNA-378 was significantly different between the three groups; the RCC group had the highest miRNA-378 level (2.41 ± 1.43) when compared with RC (1.67 ± 1.46) and healthy control (0.37 ± 0.22, p < 0.05); the miRNA-378 level in RC group was clearly higher (p < 0.01) than in the healthy control. These results suggest that high expression of miRNA-378 may be associated with renal lesions.

**Figure 1:** Comparison of miRNA-378 expressions among healthy controls, renal cyst (RC) and renal cell carcinoma (RCC) patients before surgery and six months after surgery. ^**^p < 0.01 compared with before surgery in same group; ^#^p < 0.05, compared with RC group after surgery. ξ P < 0.01 compared with healthy subjects.

### miRNA-378 expression after surgery

Six months after surgery, the expression level of miRNA-378 in the RCC and RC groups decreased significantly when compared with same group before surgery (p < 0.05). The levels decreased 53% in the RCC group and 59% in the RC group, but were still higher than in the healthy control. When compared with healthy control, the RC group had higher levels but these were not statistically different (p > 0.05), while the RCC group maintained significantly higher levels (p < 0.05), Figure 1.

### miRNA-378 expression is correlated with clinical stage and differentiation degree

We further studied the relationship between miRNA-378 expression level and clinical pathological parameters in RCC (Table 2). The results showed that miRNA-378 expression is correlated with clinical stage and differentiation degree; patients with higher clinical stage and low differentiation degrees had a much higher expression level of miRNA-378 (3.23 ± 1.44 in stage IV *vs* 0.76 ± 1.16 in stage I; 3.98 ± 1.66 in low differentiation *vs* 1.46 ± 1.18 in high differentiation degree). Levels were not correlated with patient's age (≤50 *vs* > 50), gender, surgical strategy (partial nephrectomy *vs* radical nephrectomy), and tumor diameter (≤ 2 mm *vs* > 2 mm).

**Table 2:** The relationship between miRNA-378 expression level and clinical pathological parameters in RCC patients (n = 75).

Pathological parameter	Cases	miRNA-378 (Mean ± SD)	*T* value	*P* value
Age (yr)			0.26	0.14
≤50	27	2.14 ± 0.98		
> 50	48	2.56 ± 1.22		
Gender			0.133	0.07
Male	49	1.39 ± 1.08		
Female	26	2.45 ± 1.34		
Clinical stages				
I	21	0.76 ± 1.16	−2.895	0.002
II	14	1.64 ± 1.24		
III	18	2.84 ± 1.52		
IV	12	3.23 ± 1.44		
Operation mode				
Partial nephrectomy	52	2.08 ± 1.24	0.19	0.089
Radical nephrectomy	23	3.17 ± 1.89		
Differentiation degree				
High	28	1.46 ± 1.18	−0.675	0.001
Middle	30	2.42 ± 1.24		
Low	17	3.98 ± 1.66		
Tumor diameter (mm)				
≤ 2	42	2.23 ± 1.05	2.362	0.129
> 2	33	2.64 ± 1.26		

### miRNA-378 in relapsed patients

According to the image or endoscopic examination results, we compared miRNA-378 expressions in patients with and without tumor recurrence (from blood samples of RCC patients six months after the surgery). Results showed that the patients with tumor recurrence had significantly higher miRNA-378 levels than patients without tumor recurrence (3.86 ± 2.16 *vs* 1.95 ± 1.03, *Z* = 26.26, p < 0.001).

### Diagnostic efficiency of serum miRNA-378 in RCC

We used miRNA-378 as a biological indicator for RCC patients and healthy people. As a sensitivity curve, the closer the ROC curve is to the upper left corner of the graph, the higher is the accuracy of the tested methods; when the AUC value is between 0.7 to 0.9, the method has a certain accuracy and if > 0.9, it has high accuracy. The AUC of miRNA-378 was 0.896 with a standard error of 0.025, 95% confidence interval of 0.847 to 0.945, and the AUC hypothesis testing was statistically significant (p < 0.001), Figure 2.

**Figure 2:** The AUC for diagnostic efficiency of serum miRNA-378 in renal cell carcinoma (RCC) patients.

## Discussion

miRNA genes account for about 1% of the whole genome, and they act via complementary pairing in the 3’UCR of target RNAs. miRNA binding results in the degradation of these mRNA and/or the inhibition of translation. miRNAs and their target mRNA molecules constitute a complex regulatory network, including the biological processes of cell proliferation, apoptosis, cell differentiation, development, stress response and other biological activity (Romero-Cordoba *et al.*, 2014).

miR-378 is a highly conserved miRNA that is expressed in a variety of tumors, such as liver cancer (Li *et al.*, 2013), non-small-cell lung cancer (Sun *et al.*, 2015), colorectal cancer and others (Wang *et al.*, 2015b). The abnormal expression of miRNA-378 could be involved in the development of tumors, and its expression may be used as a marker in clinical diagnosis, pathological classification and prognosis. Redova *et al.* (2012) used gene chips to screen 15 patients with RCC and 12 healthy controls, and they identified the expression levels of 667 miRNAs and verified candidate miRNAs by RT-qPCR. They concluded that miRNA-378 is highly expressed in RCC and it might serve as a biomarker for early diagnosis (Redova *et al.*, 2012). Lee *et al.* (2007) reported that miRNA-378 could inhibit the expression of *SuFu* and *Fus-1*, two tumor suppressor genes, and promote cell survival, tumor growth and angiogenesis.

Our study found that the expression of miRNA-378 was higher in RCC patients than in the benign tumor (RC) and healthy control groups. The relative expression of miRNA-378 in serum could effectively distinguish RCC patients and normal population, which is consistent with Redova's report. In addition, our research demonstrated that the expression of miRNA-378 was correlated with tumor differentiation degree and clinical stage, but not correlated with patients’ age and gender. In this study, the AUC was statistically significant, which indicates that miRNA-378 can effectively distinguish benign and malignant kidney lesions. Moreover, the relative expression of serum miRNA-378 in RCC and RC groups was significantly decreased at six months after surgery, which means that miRNA-378 could be used as a biological indicator for the curative effect in kidney lesions.

Blood samples have the advantage of being easy to obtain, noninvasive and repeatable. In addition, serum miRNAs have good stability and are is not easily affected by temperature and pH. Therefore, miRNA-378 can be used as a convenient biological indicator for the diagnosis of RCC. However, it is not clear whether the high expression of miRNA-378 in plasma is consistent with its expression in cancer tissues of RCC patients. Khella *et al.* (2012) analyzed 10 miRNA (miR-200c, miR-185, miR-34a, miR-142-3p, RNA, miR-155, miR-210, miR-224, miR-21, miR-592) in kidney mass tissues, and determined whether these were benign or malignant tumors. Their results showed that the miRNAs are closely related to hypoxia-induced stimulation and angiogenesis. (Youssef *et al.*, 2011) assessed 94 RCC specimens through qPCR methods and then genotyped and compared the results with pathologic examinations based on 900 miRNA detection results. The authors concluded that the diagnostic accuracy of miRNA in renal clear cell carcinoma was 100%, and 97% in papillary carcinoma.

On the other hand, there are also reports that serum miRNA-378 cannot be used for early diagnosis of RCC. (Hauser *et al.*, 2012) analyzed the serum miRNA-378 expression levels in RCC and normal persons through RT-PCR and concluded that circulating serum levels of miR-378 are unlikely to provide helpful diagnostic/prognostic information in RCC patients. Such inconsistent results might be caused by the following factors: inconsisten selection of reference genes; use of reagents from different companies; individual differences in the serum levels of expression of miRNA; rae, gender, and regional differences; and small numbers of patients.

Our study also has its limitations as we did not compare the miRNA-378 levels between serum and RCC (and RC) tissues. Furthermore, the study had a limited number of cases, and we did not perform a correlation analysis. However, our research provides useful data for diagnosis of RCC: we demonstrated that miRNA-378 is highly expressed in the plasma of cancer patients, it can be used to distinguish RCC patients and healthy controls, and its higher expression is correlated with higher clinical stages and low differentiation degrees. At present, the mechanism of miRNA-378 in the occurrence and development of RCC is not clearly explained. Larger samples are needed to clarify the role of miRNA-378 in the diagnosis of renal cell carcinoma, targeting therapy, curative effect evaluation and prognosis.
